The article "Stability Analysis and Optimal Control Strategies of an Echinococcosis Transmission Model" was published in 2022. Journal: Comput Math Methods Med.

# Stability Analysis and Optimal Control Strategies of an Echinococcosis Transmission Model

**DOI:** 10.1155/2022/6154866

**Published:** 2022-05-23

**Authors:** Run Yang, Jianglin Zhao, Yong Yan

**Affiliations:** Faculty of Science and Technology, Sichuan Minzu College, Kangding, China

## Abstract

This paper presents a deterministic compartmental model for echinococcosis transmission dynamics. The basic reproduction number of the model determines the existence and stability of the disease-free and disease-endemic equilibrium points. We further formulate the optimal control problem and obtain the necessary conditions to minimize the number of infected individuals and the associated costs. Numerical simulations show that optimal control strategies can significantly reduce the number of infected individuals to lower levels. Environmental disinfection may be essential for the elimination of infections. The results of this study will be beneficial for the prevention and control of echinococcosis in the Ganzi Tibetan Autonomous Prefecture and other areas of China.

## 1. Introduction

Human echinococcosis is a parasitic zoonosis caused by infection with the larval stage of the tapeworm Echinococcus. Note that more than 1 million people are affected with echinococcosis at any one time, and human echinococcosis is often expensive and complicated to treat and may require extensive surgery and prolonged drug therapy [1]. As a result, human echinococcosis poses a significant burden on patients and health care. The life cycle of Echinococcus consists of three stages: egg, larva, and adult (see [2–6]). Adults reside in the definitive hosts (mainly dogs), produce eggs that are passed in the feces, contaminate the environment (for example, water, dog's fur, vegetables, grass, and soil), and are immediately infectious. After ingestion by the intermediate host (mainly sheep, goats, and cattle), Echinococcus eggs (EEs) hatch and release six-hooked oncospheres which migrate into various organs (especially the liver and lung) and then develop into a hydatid cyst. The definitive hosts ingest the cyst-containing organs of the infected intermediate hosts and become infected. The protoscolices begin to develop into adult stages. Humans are accidental intermediate hosts because they acquire the infection in the same way as other intermediate hosts but without the biological contribution of spreading the infection to the definitive hosts. For more related knowledge about echinococcosis, please refer to [1, 2].

Wang et al. [7] developed a deterministic compartment model of echinococcosis transmission and pointed out that the strict slaughter inspection with regard to meat inspection and offal disposal, dog anthelmintics, and public health education about hygiene and dog contact could effectively reduce the spread of echinococcosis. Wu et al. [8] stressed that human inventions (deworming EEs and killing wild dogs) could be the most effective way to control the spread of echinococcosis. Rong et al. [9] showed that promoting public health education and disposing of stray dogs could significantly help control echinococcosis spreading. Hassan and Munganga [10] emphasized that treating red foxes only or disinfecting the environment alone will not be adequate to eradicate the parasite from the community, and a combination of both control strategies would be more effective in controlling the transmission of the disease in the population. Zhu et al. [11] suggested that the low evacuation rate and high mortality rate of EEs could contribute to a significant reduction in human infection cases. Furthermore, they noted that keeping humans away from EEs and enhancing treatment rates would be highly effective in preventing echinococcosis transmission in humans. Tamarozzi et al. [12] confirmed that environmental contamination, particularly through hand-to-mouth transmission, might be of primary importance from an overall appraisal of published literatures. Craig et al. [13] said that the five key elements, preventing dogs from accessing offal, treating dogs with dewormers, meat inspection, no home slaughter, and health education on hygiene and dog contact, are still valid for reducing the spread of echinococcosis today. Zhao and Yang [14] stated that optimal control strategies aimed at minimizing the number of infected individuals and the associated costs could effectively reduce the transmission of echinococcosis.

The article "Stability Analysis and Optimal Control Strategies of an Echinococcosis Transmission Model" was published in 2022. Journal: Comput Math Methods Med.

Hassan and Munganga [10] stated that the joint control is more effective than the single one. Thus, the optimal problem of control measures is a worthwhile discussion since the optimal control strategies could reduce the number of infected individuals at the lowest cost level (see [14–21] for example). Although humans are accidental intermediate hosts and do not participate in the life cycle of Echinococcus, once a person becomes infected with the disease, it will place a significant burden on their health and finances. According to [14], we will consider human infection with echinococcosis in our modeling and discuss optimal control strategies by controlling the intensity of deworming, frequency of environmental disinfection, level of strict slaughter inspection, and frequency of health education.

The rest of this paper is organized as follows. In Section 2, a dynamical model of echinococcosis transmission with control is given. A mathematical analysis of the model is presented in Section 3. The optimal control problem is formulated, and the necessary conditions are given in Section 4. Numerical simulations are shown to explore the optimal controls in Section 5. A conclusion and discussion are given in Section 6.

The article "Stability Analysis and Optimal Control Strategies of an Echinococcosis Transmission Model" was published in 2022. Journal: Comput Math Methods Med.

## 2. Model Formulation

For the dog population, the definitive hosts are divided into two classes: susceptible *S*_*d*_(*t*) and infected *I*_*d*_(*t*). For the livestock population, the intermediate hosts are decomposed into susceptible *S*_*l*_(*t*) and infected *I*_*l*_(*t*). The definitive hosts are infected by ingesting the cyst-containing organs of the infected intermediate hosts. The intermediate hosts become infected by ingesting EEs from their living environment. Humans act as accidental intermediate hosts, acquiring infection when they ingest EEs. The total human population is separated into susceptible *S*_*h*_(*t*), exposed *E*_*h*_(*t*), and infected *I*_*h*_(*t*). The EEs released from the feces of infected dogs are denoted by *X*(*t*). A schematic diagram for the dynamical transmission of echinococcosis is demonstrated in Figure 1. Based on this schematic diagram, it has the following transmission model:

(1) $$\begin{array}{c} \left\{\begin{array}{c} {\dot{S}}_{d}=\Lambda_{d}-\left(1-u_{1}\left(t\right)\right)\varepsilon \beta_{d}S_{d}I_{l}-\mu_{d}S_{d}+\delta_{d}u_{2}\left(t\right)I_{d},\\ {\dot{I}}_{d}=\left(1-u_{1}\left(t\right)\right)\varepsilon \beta_{d}S_{d}I_{l}-\mu_{d}I_{d}-\delta_{d}u_{2}\left(t\right)I_{d},\\ \dot{X}=\gamma I_{d}-\mu_{x}X-c_{h}u_{3}\left(t\right)X,\\ {\dot{S}}_{l}=\Lambda_{l}-\beta_{l}S_{l}X-\varepsilon S_{l}-\mu_{l}S_{l},\\ {\dot{I}}_{l}=\beta_{l}S_{l}X-\varepsilon I_{l}-\mu_{l}I_{l},\\ {\dot{S}}_{h}=\Lambda_{h}-\left(1-u_{4}\left(t\right)\right)\beta_{h}S_{h}X-\mu_{h}S_{h}+\delta_{h}I_{h},\\ {\dot{E}}_{h}=\left(1-u_{4}\left(t\right)\right)\beta_{h}S_{h}X-\omega E_{h}-\mu_{h}E_{h},\\ {\dot{I}}_{h}=\omega E_{h}-\mu_{h}I_{h}-\delta_{h}I_{h}. \end{array}\right. \end{array}$$

In (1), *Λ*_*d*_ denotes the annual recruitment rate of the susceptible dogs, *μ*_*d*_ is the natural death rate of the dog population, *δ*_*d*_ represents the recovery rate of infectious dogs, and *u*_2_(*t*) ∈ [0, 1] is the control on the use of praziquantel (PZQ) dosing for infected dogs. (1 − *u*_1_(*t*))*εβ*_*d*_*S*_*d*_*I*_*l*_ describes the transmission of echinococcosis between susceptible definitive hosts and infectious intermediate hosts, *u*_1_(*t*) ∈ [0, 1] is the control on the use of very strict slaughter inspection with regard to meat inspection and offal disposal for livestock, and *ε* is the home slaughter fraction of livestock. In resource-poor pastoral regions, livestock traditionally pervade home slaughter, so the dog infection rate depends on the home slaughter fraction *ε* of livestock being available for offal of infected livestock. *γ* denotes the released rate of EEs by infectious definitive hosts, *μ*_*x*_ accounts for the natural death rate of EEs, *c*_*h*_ is the death rate of EEs because of environmental disinfection, and *u*_3_(*t*) ∈ [0, 1] is the control on the use of environmental disinfection for EEs. *Λ*_*l*_ represents the annual recruitment rate of susceptible intermediate hosts, *μ*_*l*_ is the natural death rate of livestock, and *β*_*l*_*S*_*l*_*X* depicts the transmission of EEs to livestock by ingesting EEs in the environment. *Λ*_*h*_ is the annual recruitment rate of a susceptible human population, *μ*_*h*_ represents the natural death rate of humans, (1 − *u*_4_(*t*))*β*_*h*_*S*_*h*_*X* describes the transmission of echinococcosis between susceptible humans and an infectious population, and *u*_4_(*t*) is the control on the use of health education for humans. When ingesting EEs, humans are infected and then undergo an incubation period 1/*ω*. The infectious humans recover by an infectious period of mean duration 1/*δ*_*h*_.

The article "Stability Analysis and Optimal Control Strategies of an Echinococcosis Transmission Model" was published in 2022. Journal: Comput Math Methods Med.

## 3. Model Analysis

When the control variables are considered constant, some mathematical analysis results of model (1) can be obtained.

### 3.1. Positivity and Boundary of Solutions

**Theorem 1 .**

- The solution of model (1) with positive initial conditions is positive for all *t* > 0
- All positive solutions of model (1) with positive initial conditions have the upper boundary in ℝ_+_^7^

**Proof**

- Let (*S*_*d*_(*t*), *I*_*d*_(*t*), *X*(*t*), *S*_*l*_(*t*), *I*_*l*_(*t*), *S*_*h*_(*t*), *E*_*h*_(*t*), *I*_*h*_(*t*)) be a solution of model (1) with positive initial values. Define

(2) $$\begin{array}{c} t_{1}=\sup\left\{t>0:S_{d}\left(\tau \right)>0,I_{d}\left(\tau \right)>0,X\left(\tau \right)>0,S_{l}\left(\tau \right)>0,I_{l}\left(\tau \right)>0,S_{h}\left(\tau \right)>0,E_{h}\left(\tau \right)>0,I_{h}\left(\tau \right)>0\right\}, \end{array}$$

for all *τ* ∈ [0, *t*].

Since min{*S*_*d*_(0), *I*_*d*_(0), *X*(0), *S*_*l*_(0), *I*_*l*_(0), *S*_*h*_(0), *E*_*h*_(0), *I*_*h*_(0)} > 0, then there must be *t*_1_ > 0. If *t*_1_ < ∞, it gives

(3) $$\begin{array}{c} \min\left\{S_{d}\left(t_{1}\right),I_{d}\left(t_{1}\right),X\left(t_{1}\right),S_{l}\left(t_{1}\right),I_{l}\left(t_{1}\right),S_{h}\left(t_{1}\right),E_{h}\left(t_{1}\right),I_{h}\left(t_{1}\right)\right\}=0, \end{array}$$

and *S*_*d*_(*t*) > 0, *I*_*d*_(*t*) > 0, *X*(*t*) > 0, *S*_*l*_(*t*) > 0, *I*_*l*_(*t*) > 0, *S*_*h*_(*t*) > 0, *E*_*h*_(*t*) > 0, *I*_*h*_(*t*) > 0 for all *t* ∈ [0, *t*_1_).

The article "Stability Analysis and Optimal Control Strategies of an Echinococcosis Transmission Model" was published in 2022. Journal: Comput Math Methods Med.

On the other hand, the first equation of model (1) could be written as

(4) $$\begin{array}{c} \frac{d}{dt}\left[S_{d}\exp\left(\int_{0}^{t}\left(\left(1-u_{1}\right)\varepsilon \beta_{d}I_{l}+\mu_{d}\right)ds\right)\right]=\left(\Lambda_{d}+\sigma u_{2}I_{d}\right)\exp\left(\int_{0}^{t}\left(\left(1-u_{1}\right)\varepsilon \beta_{d}I_{l}+\mu_{d}\right)ds\right). \end{array}$$

Consequently,

(5) $$\begin{array}{c} S_{d}\left(t_{1}\right)=S_{d}\left(0\right)\exp\left(-\int_{0}^{t_{1}}\left(\left(1-u_{1}\right)\varepsilon \beta_{d}I_{l}+\mu_{d}\right)dt\right)+\exp\left(-\int_{0}^{t_{1}}\left(\left(1-u_{1}\right)\varepsilon \beta_{d}I_{l}+\mu_{d}\right)dt\right)\times \int_{0}^{t_{1}}\left[\left(\Lambda_{d}+\sigma u_{2}I_{d}\right)\left(\exp\left(\int_{0}^{t}\left(\left(1-u_{1}\right)\varepsilon \beta_{d}I_{l}+\mu_{d}\right)ds\right)\right)\right]dt, \end{array}$$

which implies that *S*_*d*_(*t*_1_) > 0. A similar approach could be applied to show that *I*_*d*_(*t*_1_) > 0, *S*_*l*_(*t*_1_) > 0, *I*_*l*_(*t*_1_) > 0 and *E*(*t*_1_) > 0, which is a contradiction. Therefore, *t*_1_ = ∞.

Hence, all solutions of model (1) with positive initial conditions remain positive when *t* > 0.

(ii) The first two equations of model (1) could be transformed into

(6) $$\begin{array}{c} \frac{d\left(S_{d}+I_{d}\right)}{dt}=\Lambda_{d}-\mu_{d}\left(S_{d}+I_{d}\right)\leq \Lambda_{d}-\mu_{d}\left(S_{d}+I_{d}\right). \end{array}$$

Thus, $\underset{t⟶\infty }{\text{limsup}}\left(S_{d}+I_{d}\right)\leq \Lambda_{d}/\mu_{d}$.

The fourth and fifth equations of model (1) could be transformed into

(7) $$\begin{array}{c} \frac{d\left(S_{l}+I_{l}\right)}{dt}=\Lambda_{l}-\left(\mu_{l}+\varepsilon \right)\left(S_{l}+I_{l}\right)\leq \Lambda_{l}-\left(\mu_{l}+\varepsilon \right)\left(S_{l}+I_{l}\right), \end{array}$$

which leads to $\underset{t⟶\infty }{\text{limsup}}\left(S_{l}+I_{l}\right)\leq \Lambda_{l}/\left(\mu_{l}+\varepsilon \right)$.

The last three equations of model (1) give

(8) $$\begin{array}{c} \frac{d\left(S_{h}+E_{h}+I_{h}\right)}{dt}=\Lambda_{h}-\mu_{h}\left(S_{h}+E_{h}+I_{h}\right)\leq \Lambda_{h}-\mu_{h}\left(S_{h}+E_{h}+I_{h}\right), \end{array}$$

which yields $\underset{t⟶\infty }{\text{limsup}}\left(S_{h}+E_{h}+I_{h}\right)\leq \Lambda_{h}/\mu_{h}$.

From the third equation of model (1), there is

(9) $$\begin{array}{c} \frac{dX}{dt}=\gamma I_{d}-\left(\mu_{x}+c_{h}u_{3}\right)X\leq \frac{\gamma \Lambda_{d}}{\mu_{d}}-\left(\mu_{x}+c_{h}u_{3}\right)X. \end{array}$$

Hence, $\underset{t⟶\infty }{\text{limsup}}X\leq \gamma \Lambda_{d}/\mu_{d}\left(\mu_{x}+c_{h}u_{3}\right)$.

Let

(10) $$\begin{array}{c} \Gamma =\left\{\left(S_{d},I_{d},E,S_{d},I_{d},S_{h},I_{h}\right)\in {\mathbb{R}}_{+}^{7}:S_{d}+I_{d}\leq \frac{\Lambda_{d}}{\mu_{d}},X\leq \frac{\gamma \Lambda_{d}}{\mu_{d}\left(\mu_{e}+c_{h}u_{3}\right)},S_{l}+I_{l}\leq \frac{\Lambda_{l}}{\mu_{l}+\varepsilon },S_{h}+E_{h}+I_{h}\leq \frac{\Lambda_{h}}{\mu_{h}}\right\}. \end{array}$$

Thus, all positive solutions of model (1) with positive initial conditions ultimately have the upper boundary in ℝ_+_^7^. The closed set Γ is positively invariant and attracts the solution to model (1).

The article "Stability Analysis and Optimal Control Strategies of an Echinococcosis Transmission Model" was published in 2022. Journal: Comput Math Methods Med.

### 3.2. Equilibrium Points and Stability Analysis

In this section, some mathematical analysis results of model (1) can be obtained when the controls are supposed to be constant.

The disease-free equilibrium of model (1) is denoted by

(11) $$\begin{array}{c} E_{dfe}=\left(S_{d}^{0},0,0,S_{l}^{0},0,S_{h}^{0},0,0\right)=\left(\frac{\Lambda_{d}}{\mu_{d}},0,0,\frac{\Lambda_{l}}{\varepsilon +\mu_{l}},0,\frac{\Lambda_{h}}{\mu_{h}},0,0\right). \end{array}$$

In the next, the next-generation matrix approach [22] will be applied for computing the basic reproduction number *ℛ*_0_. The matrix of new infection *ℱ* and the matrix of transition *𝒱* are defined as follows:

(12) $$\begin{array}{c} F=\left[\begin{array}{c} \left(1-u_{1}\right)\varepsilon \beta_{d}S_{d}I_{l}\\ \gamma I_{d}\\ \beta_{l}S_{l}X\\ \left(1-u_{4}\right)\beta_{h}S_{h}X\\ 0 \end{array}\right],V=\left[\begin{array}{c} \left(\mu_{d}+\delta_{d}u_{2}\right)I_{d}\\ \left(\mu_{x}+c_{h}u_{3}\right)X\\ \left(\varepsilon +\mu_{l}\right)I_{l}\\ \left(\omega +\mu_{h}\right)E_{h}\\ -\omega E_{h}+\left(\mu_{h}+\delta_{h}\right)I_{h} \end{array}\right]. \end{array}$$

Furthermore, the Jacobian matrices of *ℱ* and *𝒱* at the disease-free equilibrium *E*_*dfe*_ are, respectively, obtained by

(13) $$\begin{array}{c} F=\left[\begin{array}{ccccc} 0 & 0 & \frac{\left(1-u_{1}\right)\varepsilon \beta_{d}\Lambda_{d}}{\mu_{d}} & 0 & 0\\ \gamma & 0 & 0 & 0 & 0\\ 0 & \frac{\beta_{l}\Lambda_{l}}{\varepsilon +\mu_{l}} & 0 & 0 & 0\\ 0 & \frac{\left(1-u_{4}\right)\beta_{h}\Lambda_{h}}{\mu_{h}} & 0 & 0 & 0\\ 0 & 0 & 0 & 0 & 0 \end{array}\right],V=\left[\begin{array}{ccccc} \mu_{d}+\delta_{d}u_{2} & 0 & 0 & 0 & 0\\ 0 & \mu_{x}+c_{h}u_{3} & 0 & 0 & 0\\ 0 & 0 & \varepsilon +\mu_{l} & 0 & 0\\ 0 & 0 & 0 & \omega +\mu_{h} & 0\\ 0 & 0 & 0 & -\omega & \mu_{h}+\delta_{h} \end{array}\right]. \end{array}$$

Then, the basic reproduction number that is the largest eigenvalue with a large domain of the next generation matrix *FV*^−1^ is given by

(14) $$\begin{array}{c} R_{0}=\sqrt[{3}]{R_{0x}\cdot R_{0d}\cdot R_{0l}}, \end{array}$$

where

(15) $$\begin{array}{c} R_{0x}=\frac{\gamma }{\mu_{x}+c_{h}u_{3}},R_{0d}=\frac{1}{\mu_{d}+\delta_{d}u_{2}}\cdot \frac{\Lambda_{d}}{\mu_{d}}\cdot \left(1-u_{1}\right)\varepsilon \beta_{d},R_{0l}=\frac{1}{\varepsilon +\mu_{l}}\cdot \frac{\Lambda_{l}}{\varepsilon +\mu_{l}}\cdot \beta_{l}. \end{array}$$

Here, *ℛ*_0*x*_ denotes the average number of EEs that might be ingested by the intermediate host livestock and humans, *ℛ*_0*d*_ describes the average number of infected dogs by infected livestock, and *ℛ*_0*l*_ accounts for the average number of infected livestock by EEs. For more ecological and epidemiological significance in (14), please refer to [7, 8, 22].

The article "Stability Analysis and Optimal Control Strategies of an Echinococcosis Transmission Model" was published in 2022. Journal: Comput Math Methods Med.

Assume that *E*_*ee*_ = (*S*_*d*_^∗^, *I*_*d*_^∗^, *X*^∗^, *S*_*l*_^∗^, *I*_*l*_^∗^, *S*_*h*_^∗^, *E*_*h*_^∗^, *I*_*h*_^∗^) should be the endemic equilibrium of model (1). Let the right-hand sides of model (1) vanish. By solving these equations, it gives

(16) $$\begin{array}{c} S_{d}^{*}=\frac{\left(\mu_{d}+\delta_{d}u_{2}\right)I_{d}^{*}}{\left(1-u_{1}\right)\varepsilon \beta_{d}I_{l}^{*}},I_{d}^{*}=\frac{\mu_{e}+c_{h}u_{3}}{\gamma }X^{*},S_{l}^{*}=\frac{\Lambda_{l}}{\beta_{l}X^{*}+\varepsilon +\mu_{l}},\\ I_{l}^{*}=\frac{\beta_{l}S_{l}^{*}X^{*}}{\varepsilon +\mu_{l}},X^{*}=\frac{\left(\mu_{d}+\delta_{d}u_{2}\right){\left(\varepsilon +\mu_{l}\right)}^{2}}{\beta_{l}\left[\left(\mu_{d}+\delta_{d}u_{2}\right)\left(\varepsilon +\mu_{l}\right)+\left(1-u_{1}\right)\varepsilon \beta_{d}\Lambda_{l}\right]}\left(R_{0}^{3}-1\right),\\ S_{h}^{*}=\frac{\left(\omega +\mu_{h}\right)E_{h}^{*}}{\left(1-u_{4}\right)\beta_{h}X^{*}},I_{h}^{*}=\frac{\omega E_{h}^{*}}{\mu_{h}+\delta_{h}},\\ E_{h}^{*}=\frac{\left(1-u_{4}\right)\beta_{h}X^{*}\left(\mu_{h}+\delta_{h}\right)\Lambda_{h}}{\mu_{h}\left[\left(\omega +\mu_{h}\right)\left(\mu_{h}+\delta_{h}\right)+\left(1-u_{4}\right)\beta_{h}X^{*}\left(\omega +\mu_{h}+\delta_{h}\right)\right]}. \end{array}$$

Then, it is clear that model (1) has a uniquely endemic equilibrium *E*_*ee*_ if and only if *ℛ*_0_ > 1.

A similar method from [7, 9] is used to obtain the following results. Appendix A gives the detailed proof of Theorem 2. In Appendix B, the proof of Theorem 3 is presented. The proof of Theorem 4 can be displayed in Appendix C.

**Theorem 2 .**

The disease-free equilibrium *E*_*dfe*_ is locally asymptotically stable if *ℛ*_0_ < 1 and is unstable if *ℛ*_0_ > 1.

**Theorem 3 .**

The disease-free equilibrium *E*_*dfe*_ is globally asymptotically stable if *ℛ*_0_ < 1.

**Theorem 4 .**

The uniquely endemic equilibrium *E*_*ee*_ of model (1) is globally asymptotically stable when *ℛ*_0_ > 1.

## 4. Optimal Control

To obtain the optimal control strategies, an objective functional is defined by

(17) $$\begin{array}{c} J\left(u\right)=\int_{0}^{T}g\left(\phi ,u,t\right)dt=\int_{0}^{T}\left[I_{d}+I_{l}+I_{h}+\frac{1}{2}\left(c_{1}u_{1}^{2}+c_{2}u_{2}^{2}+c_{3}u_{3}^{2}+c_{4}u_{4}^{2}\right)\right]dt, \end{array}$$

subject to the state system (1). *ϕ* = (*S*_*d*_, *I*_*d*_, *X*, *S*_*l*_, *I*_*l*_, *S*_*h*_, *E*_*h*_, *I*_*h*_) is the solution of model (1) with positive initial values and **u** = (*u*_1_(*t*), *u*_2_(*t*), *u*_3_(*t*), *u*_4_(*t*)). *c*_1_, *c*_2_, *c*_3_, and *c*_4_ represent the weight constants of the control variables *u*_1_, *u*_2_, *u*_3_, and *u*_4_, respectively. (1/2)*c*_1_*u*_1_^2^, (1/2)*c*_2_*u*_2_^2^, (1/2)*c*_3_*u*_3_^2^, and (1/2)*c*_4_*u*_4_^2^ denote the costs of home slaughter inspection, anthelmintic treatment, environmental disinfection, and health education, respectively.

The article "Stability Analysis and Optimal Control Strategies of an Echinococcosis Transmission Model" was published in 2022. Journal: Comput Math Methods Med.

The objective of the optimal control problem (17) is to find a control set that minimizes the infected dogs, the infected livestock, and the infected humans when minimizing the control cost function. Let **U** = {**u** = (*u*_1_(*t*), *u*_2_(*t*), *u*_3_(*t*), *u*_4_(*t*)): 0 ≤ *u*_*i*_(*t*) ≤ 1, *t* ∈ [0, *T*], *i* = 1, 2, 3, 4} be a measurable set. Then, there needs to be the optimal control **u**^∗^ = (*u*_1_^∗^(*t*), *u*_2_^∗^(*t*), *u*_3_^∗^(*t*), *u*_4_^∗^(*t*)) such that

(18) $$\begin{array}{c} J\left(u^{*}\right)=\min\left\{J\left(u\right)\text{: }u\in U\right\}. \end{array}$$

The necessary conditions that determine the optimal control **u**^∗^ satisfying (5) with constraint model (1) are derived from Pontryagin's Maximum Principle. Then, the optimal control problem (18) is transformed into minimizing the following Hamiltonian function:

(19) $$\begin{array}{c} H=g\left(\phi ,u,t\right)+\overset{8}{\underset{i=1}{\sum }}\lambda_{i}f_{i}\left(\phi ,u,t\right), \end{array}$$

where *f*_*i*_(*ϕ*, **u**, *t*), *i* = 1, 2, 3, 4, 5, 6, 7, 8, are the right-hand sides of model (1). And *λ*_*i*_, *i* = 1, 2, 3, 4, 5, 6, 7, 8, are the adjoint variables that satisfy the following costate system:

(20) $$\begin{array}{c} \left\{\begin{array}{c} {\dot{\lambda }}_{1}=-\frac{\partial H}{\partial S_{d}}=\left(1-u_{1}\right)\varepsilon \beta_{d}I_{l}\left(\lambda_{1}-\lambda_{2}\right)+\lambda_{1}\mu_{d},\\ {\dot{\lambda }}_{2}=-\frac{\partial H}{\partial I_{d}}=-1-\lambda_{1}\delta_{d}u_{2}+\lambda_{2}\left(\mu_{d}+\delta_{d}u_{2}\right)-\lambda_{3}\gamma ,\\ {\dot{\lambda }}_{3}=-\frac{\partial H}{\partial X}=\lambda_{3}\left(\mu_{x}+c_{h}u_{3}\right)+\left(\lambda_{4}-\lambda_{5}\right)\beta_{l}S_{l}+\left(\lambda_{6}-\lambda_{7}\right)\left(1-u_{4}\right)\beta_{h}S_{h},\\ {\dot{\lambda }}_{4}=-\frac{\partial H}{\partial S_{l}}=\lambda_{4}\left(\beta_{l}X+\varepsilon +\mu_{l}\right)-\lambda_{5}\beta_{l}X,\\ {\dot{\lambda }}_{5}=-\frac{\partial H}{\partial I_{l}}=-1+\left(1-u_{1}\right)\varepsilon \beta_{d}S_{d}\left(\lambda_{1}-\lambda_{2}\right)+\lambda_{5}\left(\mu_{l}+\varepsilon \right),\\ {\dot{\lambda }}_{6}=-\frac{\partial H}{\partial S_{h}}=\left(1-u_{4}\right)\beta_{h}X\left(\lambda_{6}-\lambda_{7}\right)+\lambda_{6}\mu_{h},\\ {\dot{\lambda }}_{7}=-\frac{\partial H}{\partial E_{h}}=\lambda_{7}\left(\omega +\mu_{h}\right)-\lambda_{8}\omega ,\\ {\dot{\lambda }}_{8}=-\frac{\partial H}{\partial I_{h}}=-1-\lambda_{6}\delta_{h}+\lambda_{8}\left(\delta_{h}+\mu_{h}\right), \end{array}\right. \end{array}$$

with boundary conditions *λ*_*i*_(*T*) = 0, *i* = 1, 2, 3, 4, 5, 6, 7, 8. Additionally, the optimality conditions *∂H*/*∂u*_*i*_ = 0, *i* = 1, 2, 3, 4, lead to the optimal controls:

(21) $$\begin{array}{c} u_{i}^{*}=\min\left\{1,\max\left\{0,u_{i}^{c}\right\}\right\},\;i=1,2,3,4, \end{array}$$

where

(22) $$\begin{array}{c} u_{1}^{c}=\frac{\varepsilon \beta_{d}S_{d}I_{l}\left(\lambda_{2}-\lambda_{1}\right)}{c_{1}},u_{2}^{c}=\frac{\delta_{d}I_{d}\left(\lambda_{2}-\lambda_{1}\right)}{c_{2}},u_{3}^{c}=\frac{\lambda_{3}c_{h}X}{c_{3}},u_{4}^{c}=\frac{\left(\lambda_{7}-\lambda_{6}\right)\beta_{h}S_{h}X}{c_{4}}. \end{array}$$

The article "Stability Analysis and Optimal Control Strategies of an Echinococcosis Transmission Model" was published in 2022. Journal: Comput Math Methods Med.

## 5. Numerical Simulations

In this section, the numerical results of different optimal control scenarios *u*_1_, *u*_2_, *u*_3_, and *u*_4_ are presented. The numerical solution of the optimality system is solved by the forward-backward sweep method [27]. The ode45 solver in MATLAB is used to solve (1) with initial values *S*_*d*_(0) = 1.686 × 10^5^, *I*_*d*_(0) = 4 × 10^4^, *S*_*l*_(0) = 3.335 × 10^6^, *I*_*l*_(0) = 5 × 10^5^, *X*(0) = 2 × 10^7^, *S*_*h*_(0) = 8.05 × 10^5^, *E*_*h*_(0) = 8.064 × 10^3^, and *I*_*h*_(0) = 576, where *S*_*d*_(0) can be estimated from [28] and *S*_*l*_(0), *S*_*h*_(0), *I*_*h*_(0) can be estimated from [30]. The other initial values of model (1) are assumed. The costate system (20) with boundary conditions *λ*_*i*_(*T*) = 0, *i* = 1, 2, 3, 4, 5, 6, 7, 8, is numerically obtained from the backward Runge-Kutta scheme. The control variables (21) are updated by entering the new state and adjoint values until the current state; the adjoint and control values are negligibly close. It is well established that the cost of anthelmintic treatment is more expensive than that of environmental disinfection, while the cost of slaughter inspection is cheaper than that of environmental disinfection. On the other hand, the cost of health education is cheaper than that of slaughter inspection. Hence, the weighting constants are considered as *c*_1_ = 50, *c*_2_ = 90, *c*_3_ = 70, and *c*_4_ = 60. All other parameters are listed in Table 1. *Λ*_*l*_ is estimated by using the data from the Statistics Bureau of Ganzi Tibetan Autonomous Prefecture [28]. *Λ*_*d*_, *ε*, *δ*_*d*_, and *δ*_*h*_ are estimated by using the data from Zou [30]. The average life expectancy of people in Ganzi Tibetan Autonomous Prefecture (see [29]) was 72.10 years in 2016. Therefore, the natural death rate *μ*_*h*_ of humans in Ganzi Tibetan Autonomous Prefecture is estimated as *μ*_*h*_ = 1/72.1 ≈ 0.0139. The death rate of echinococcosis eggs due to environmental disinfection cannot be directly acquired. It is instead assumed that the parasite egg mortality rate induced by environmental disinfection should arrive at ten times higher than the natural death rate. The combined employment of two, three, and four control measures will be studied. The following scenarios are considered:

(A) *Scenario one*: coupled control measures
  - *Strategy A*: slaughter inspection and anthelmintic treatment (*u*_1_, *u*_2_)
  - *Strategy B*: slaughter inspection and environmental disinfection (*u*_1_, *u*_3_)
  - *Strategy C*: slaughter inspection and health education (*u*_1_, *u*_4_)
  - *Strategy D*: anthelmintic treatment and environmental disinfection (*u*_2_, *u*_3_)
  - *Strategy E*: anthelmintic treatment and health education (*u*_2_, *u*_4_)
  - *Strategy F*: environmental disinfection and health education (*u*_3_, *u*_4_)
(B) *Scenario two*: threefold control measures
  - *Strategy G*: slaughter inspection, anthelmintic treatment, and environmental disinfection (*u*_1_, *u*_2_, *u*_3_)
  - *Strategy H*: slaughter inspection, anthelmintic treatment, and health education (*u*_1_, *u*_2_, *u*_4_)
  - *Strategy I*: slaughter inspection, environmental disinfection, and health education (*u*_1_, *u*_3_, *u*_4_)
  - *Strategy J*: anthelmintic treatment, environmental disinfection, and health education (*u*_2_, *u*_3_, *u*_4_
(C) *Scenario three*: fourfold control measures
  - *Strategy K*: slaughter inspection, anthelmintic treatment, environmental disinfection, and health education (*u*_1_, *u*_2_, *u*_3_, *u*_4_)

For Strategy A, the slaughter inspection control *u*_1_ and the anthelmintic treatment control *u*_2_ are merely carried out while the environmental disinfection control *u*_3_ and the health education control *u*_4_ are chosen to be ignored.  Figure 2(a) shows the paths of optimal controls *u*_1_^∗^ and *u*_2_^∗^. The slaughter inspection (blue dash-dot line in Figure 2(a)) should be executed 100% for 15 years and then decreases gradually to zero. Meanwhile, the anthelmintic treatment (red dotted line in Figure 2(a)) needs to start the 100% use for 10 years and then declines to zero. Figures 2(b)–2(d) illustrates the effect of the optimal controls *u*_1_^∗^ and *u*_2_^∗^. When there is no control (see the blue dashed lines in Figures 2(b)–2(d)), the disease is prevalent. However, when the optimal controls are implemented (see the red dotted lines in Figures 2(b)–2(d)), the number of infected dogs, infected livestock, and infected humans could be significantly minimized to the lower level (*I*_*d*_, *I*_*l*_, *I*_*h*_) = (61,207,6). For Strategy B, the slaughter inspection control *u*_1_ and the environmental disinfection control *u*_3_ are merely applied in (17) while the anthelmintic treatment and health education are not considered, i.e., *u*_2_ = 0, *u*_4_ = 0.  Figure 3(a) presents the profiles of optimal controls *u*_1_^∗^ and *u*_3_^∗^. The slaughter inspection (blue dash-dot line in Figure 3(a)) is done 100% intensively for 16 years and then decreases gradually till the end of control. Meanwhile, the environmental disinfection control (green dash-dot line in Figure 3(a)) begins with 100% use for 32 years and then declines to zero. Figures 3(b)–3(d) display the effect of *u*_1_^∗^ and *u*_3_^∗^. It is obvious that there is a considerable difference in the number of infected dogs, infected livestock, and infected humans between the controlled cases (see the blue dashed lines in Figures 3(b)–3(d)) and the cases without control (see the red dotted lines in Figures 3(b)–3(d)). The number of infected dogs, infected livestock, and infected humans under Strategy B could drop to the lower level (*I*_*d*_, *I*_*l*_, *I*_*h*_) = (24,61,6). For Strategy C, *u*_1_ and *u*_4_ are merely considered in (17) while *u*_2_ and *u*_3_ are ignored.  Figure 4(a) shows the profiles of optimal controls *u*_1_^∗^ and *u*_4_^∗^. The slaughter inspection (blue dash-dot line in Figure 4(a)) is kept at the maximum use of 100% for 34 years and then declines gradually to zero. On the contrary, the health education *u*_4_^∗^ (black dashed line in Figure 4(a)) declines from the maximum use of 46.1% to zero in 16 years. Figures 4(b)–4(d) display that the number of infected dogs, infected livestock, and infected humans could drop to the lower level (*I*_*d*_, *I*_*l*_, *I*_*h*_) = (319,1070,8). For Strategy D, *u*_2_ and *u*_3_ are implemented to optimize the objective functional (17) while *u*_1_ = 0 and *u*_4_ = 0.  Figure 5(a) shows the paths of *u*_2_^∗^ and *u*_3_^∗^. Both the anthelmintic treatment (red dotted line in Figure 5(a)) and the environmental disinfection (green dash-dot line in Figure 5(a)) should be done 100% intensively for 14 years and then decline gradually to zero. Figures 5(b)–5(d) display that there could exist a considerable significance for reducing the number of infected dogs, infected livestock, and infected humans (blue dashed line) that drops to the lower level (*I*_*d*_, *I*_*l*_, *I*_*h*_) = (6,16,5). For Strategy E, *u*_2_ and *u*_4_ are considered while *u*_1_ = 0 and *u*_3_ = 0.  Figure 6(a) shows the profiles of *u*_2_^∗^ and *u*_4_^∗^. The control *u*_2_^∗^ (red dotted line in Figure 6(a)) has a 100% use for 25 years and then drops gradually to zero. Meanwhile, the control effort *u*_4_^∗^ (black dashed line in Figure 6(a)) decays from the maximum use of 46.1% to zero in 14 years. Figures 6(b)–6(d) suggest that Strategy E could provide a significant reduction in the number of infected dogs, infected livestock, and infected humans that decreases to the lower level (*I*_*d*_, *I*_*l*_, *I*_*h*_) = (118,396,7). For Strategy F, *u*_3_ and *u*_4_ are considered while *u*_1_ = 0 and *u*_2_ = 0.  Figure 7(a) presents the paths of *u*_3_^∗^ and *u*_4_^∗^. The control *u*_3_^∗^ (green dash-dot line in Figure 7(a)) needs to perform a 100% use for 39 years and then gradually decreases to zero. Meanwhile, the control *u*_4_^∗^ (black dashed line in Figure 7(a)) drops rapidly from the maximum use of 46.1% to zero in five years. Figures 7(b)–7(d) show that Strategy F could provide a significant reduction in the number of infected dogs, infected livestock, and infected humans that drops to the lower level (*I*_*d*_, *I*_*l*_, *I*_*h*_) = (35,84,6).

The article "Stability Analysis and Optimal Control Strategies of an Echinococcosis Transmission Model" was published in 2022. Journal: Comput Math Methods Med.

For Strategy G, the controls *u*_1_, *u*_2_, and *u*_3_ are considered while *u*_4_ = 0.  Figure 8(a) shows the paths of *u*_1_^∗^, *u*_2_^∗^, and *u*_3_^∗^. The control *u*_1_^∗^ (blue dash-dot line in Figure 8(a)) has a 100% use for 12 years and then decreases gradually to zero. Both the control *u*_2_^∗^ (red dotted line in Figure 8(a)) and the control *u*_3_^∗^ (green dash-dot line in Figure 8(a)) have a 100% use for 10 years and then drop gradually to zero. Figures 8(b)–8(d) suggest that the number of infected dogs, infected livestock, and infected humans under Strategy G (blue dashed line) could be significantly reduced to a lower level (*I*_*d*_, *I*_*l*_, *I*_*h*_) = (6,15,5) compared to no control (red dotted line). For Strategy H, the controls *u*_1_, *u*_2_, and *u*_4_ are considered while *u*_3_ = 0.  Figure 9(a) presents the paths of *u*_1_^∗^, *u*_2_^∗^, and *u*_4_^∗^. The slaughter inspection (blue dash-dot line in Figure 9(a)) should be done 100% for 15 years and then decreases gradually to zero. The anthelmintic treatment *u*_2_^∗^ (red dotted line in Figure 9(a)) has the 100% use for 10 years and then declines to zero. On the contrary, the health education *u*_4_^∗^ (black dashed line in Figure 9(a)) drops rapidly from the maximum use of 46.1% to zero in 11 years. Figures 9(b)–9(d) display that there is a significance for *u*_1_^∗^, *u*_2_^∗^, and *u*_4_^∗^ reducing the number of infected dogs, infected livestock, and infected humans (blue dashed line) that drops to a lower level (*I*_*d*_, *I*_*l*_, *I*_*h*_) = (62,207,6). For Strategy I, *u*_1_, *u*_3_, and *u*_4_ are implemented in (17) while *u*_2_ = 0.  Figure 10(a) shows the paths of *u*_1_^∗^, *u*_3_^∗^, and *u*_4_^∗^. The control *u*_1_^∗^ (blue dash-dot line in Figure 10(a)) should be done 100% intensively for 16 years and then declines gradually to zero, while the control *u*_3_^∗^ (green dash-dot line in Figure 10(a)) has the maximum use (100%) for 32 years before dropping gradually to zero. The control *u*_4_^∗^ drops rapidly from the maximum use (46.1%) to zero in five years. Figures 10(b)–10(d) suggest that there could be a considerable significance for reducing the number of infected dogs, infected livestock, and infected humans (blue dashed line) that decreases to a lower level (*I*_*d*_, *I*_*l*_, *I*_*h*_) = (24,61,6). For Strategy J, *u*_2_, *u*_3_, and *u*_4_ are considered while *u*_1_ = 0. The optimal controls *u*_2_^∗^, *u*_3_^∗^, and *u*_4_^∗^ are presented in Figure 11(a). Both *u*_2_^∗^ (red dotted line in Figure 11(a)) and *u*_3_^∗^ (green dash-dot line in Figure 11(a)) have a 100% use for 14 years and then drop gradually to zero. Meanwhile, *u*_4_^∗^ (black dashed line in Figure 11(a)) drops rapidly from the maximum use of 46.1% to zero in four years. Figures 11(b)–11(d) show that Strategy J (blue dashed line) could provide a significant reduction in the number of infected dogs, infected livestock, and infected humans that deceases to the lower level (*I*_*d*_, *I*_*l*_, *I*_*h*_) = (6,16,5).

The article "Stability Analysis and Optimal Control Strategies of an Echinococcosis Transmission Model" was published in 2022. Journal: Comput Math Methods Med.

For Strategy K, all the controls *u*_1_, *u*_2_, *u*_3_, and *u*_4_ are considered in (17). The optimal controls *u*_1_^∗^, *u*_2_^∗^, *u*_3_^∗^, and *u*_4_^∗^ are displayed in Figure 12(a). The control *u*_1_^∗^ (blue dash-dot line in Figure 11(a)) starts to have a 100% use for 12 years and then decreases gradually to zero. Both the control *u*_2_^∗^ (red dotted line in Figure 11(a)) and the control *u*_3_^∗^ (green dash-dot line in Figure 12(a)) have a 100% use for 10 years and then decline gradually to zero. Meanwhile, the control *u*_4_^∗^ (black dashed line in Figure 12(a)) drops rapidly from the maximum use of 46.1% to zero in four years. Figures 12(b)–12(d) show that Strategy K (blue dashed line) has a significant reduction in the number of infected dogs, infected livestock, and infected humans that could drop to the lower level (*I*_*d*_, *I*_*l*_, *I*_*h*_) = (6,15,5).

## 6. Conclusion and Discussion

This paper presents and analyzes a deterministic compartmental system for echinococcosis transmission dynamics under the intervention of constant slaughter inspection, anthelmintic treatment, environmental disinfection, and health education. The existence and stability of the disease-free and disease-endemic equilibrium points of the model are discussed. It finds that the basic reproduction number determines entirely whether the disease is extinct or not endemic. In the absence of control measures, the basic reproduction number in Ganzi Tibetan Autonomous Prefecture is estimated to be *ℛ*_0_ = 1.0662 > 1. This means that echinococcosis is an endemic disease. Craig et al. [13] stated that it is difficult to eliminate the spread of echinococcosis in scattered seminomadic remote communities, even if the Echinococcosis Control Program in Western China is carried out by using PZQ for the dog-dosing frequency monthly. Therefore, comprehensive interventions mainly including slaughter inspection, anthelmintic treatment, environmental disinfection, and health education should be taken into account to control the transmission of echinococcosis. Figures 2–12 have shown that the optimal strategies from Strategy A to Strategy K have a considerable significance in reducing the number of infected dogs, infected livestock, and infected humans. The combined prevention and control measures could eliminate the prevalence of echinococcosis.

The article "Stability Analysis and Optimal Control Strategies of an Echinococcosis Transmission Model" was published in 2022. Journal: Comput Math Methods Med.

Note that Strategies D, G, J, and K could reduce the number of infected dogs, infected livestock, and infected humans to a lower level than other strategies. Therefore, anthelmintic treatment and environmental disinfection may play a crucial role in controlling the number of infectious individuals. The anthelmintic treatment against echinococcosis does not eliminate the infection, and most of the time, when the treatments cease, there is a rebound in the infection (see [13]). Environmental disinfection may hence be indispensable for the prevention and control of echinococcosis. However, the importance of environmental disinfection for the prevention and control of echinococcosis is often ignored. Therefore, deworming and environmental disinfection should be the primary consideration in choosing control measures when developing an echinococcosis control and prevention program. The slaughter inspection with regard to meat inspection and offal disposal is aimed at reducing the number of infected dogs. Consequently, the number of EEs naturally decreases when the slaughter inspection is implemented. Thus, infected livestock would be reduced. From this perspective, the slaughter inspection may shorten the control time. The health education is aimed at reducing the possibility of ingestion by humans. The low evacuation rate of EEs would lead to the small possibility of ingestion by humans. Therefore, if the number of EEs drops to a certain level, the health education will become unimportant. That is to say that the health education has effectiveness in a short time for the prevention and control of echinococcosis. Hence, for faster and better prevention and control of echinococcosis, Strategy K may be recommended to be implemented in the real situation. Finally, some parameter values (for example, the death rate of EEs due to environmental disinfection) are not directly available; our model does not necessarily reflect the true picture of the prevalence of echinococcosis in the Ganzi Tibetan Autonomous Prefecture. Nevertheless, our model analysis suggests that environmental disinfection is critical to controlling the spread of echinococcosis and that the optimal integrated control strategy (Strategy K) can control the disease in the shortest possible time.

The article "Stability Analysis and Optimal Control Strategies of an Echinococcosis Transmission Model" was published in 2022. Journal: Comput Math Methods Med.

## Figures and Tables

**Figure 1:** Schematic diagram of the transmission dynamics of Echinococcus.

**Figure 2:** Simulation results for Strategy A: (a) depicts the profiles of optimal controls *u*_1_^∗^ and *u*_2_^∗^; (b–d) represent the number of infected dogs, infected livestock, and infected humans, respectively.

**Figure 3:** Simulation results for Strategy B: (a) depicts the profiles of optimal controls *u*_1_^∗^ and *u*_3_^∗^; (b–d) represent the number of infected dogs, infected livestock, and infected humans, respectively.

**Figure 4:** Simulation results for Strategy C: (a) depicts the profiles of optimal controls *u*_1_^∗^ and *u*_4_^∗^; (b–d) represent the number of infected dogs, infected livestock, and infected humans, respectively.

**Figure 5:** Simulation results for Strategy D: (a) depicts the profiles of optimal controls *u*_2_^∗^ and *u*_3_^∗^; (b–d) represent the number of infected dogs, infected livestock, and infected humans, respectively.

**Figure 6:** Simulation results for Strategy E: (a) depicts the profiles of optimal controls *u*_2_^∗^ and *u*_4_^∗^; (b–d) represent the number of infected dogs, infected livestock, and infected humans, respectively.

**Figure 7:** Simulation results for Strategy F: (a) depicts the profiles of optimal controls *u*_3_^∗^ and *u*_4_^∗^; (b–d) represent the number of infected dogs, infected livestock, and infected humans, respectively.

**Figure 8:** Simulation results for Strategy G: (a) depicts the profiles of optimal controls *u*_1_^∗^, *u*_2_^∗^, and *u*_3_^∗^; (b–d) represent the number of infected dogs, infected livestock, and infected humans, respectively.

The article "Stability Analysis and Optimal Control Strategies of an Echinococcosis Transmission Model" was published in 2022. Journal: Comput Math Methods Med.

**Figure 9:** Simulation results for Strategy H: (a) depicts the profiles of optimal controls *u*_1_^∗^, *u*_2_^∗^, and *u*_4_^∗^; (b–d) represent the number of infected dogs, infected livestock, and infected humans, respectively.

**Figure 10:** Simulation results for Strategy I: (a) depicts the profiles of optimal controls *u*_1_^∗^, *u*_3_^∗^, and *u*_4_^∗^; (b–d) represent the number of infected dogs, infected livestock, and infected humans, respectively.

**Figure 11:** Simulation results for Strategy J: (a) depicts the profiles of optimal controls *u*_2_^∗^, *u*_3_^∗^, and *u*_4_^∗^; (b–d) represent the number of infected dogs, infected livestock, and infected humans, respectively.

**Figure 12:** Simulation results for Strategy K: (a) depicts the profiles of optimal controls *u*_1_^∗^, *u*_2_^∗^, *u*_3_^∗^, and *u*_4_^∗^; (b–d) represent the number of infected dogs, infected livestock, and infected humans, respectively.

**Table 1:** Description of parameters of model (1).

Parameters	Interpretation	Units	Source
*Λ*_*d*_	Recruitment rate of dogs	21.1 × 10^4^ year^−1^	Estimated
*β*_*d*_	Transmission rate from livestock to dogs	5.8 × 10^−8^ year^−1^	[7]
*μ*_*d*_	Natural death rate of dogs	0.08 year^−1^	[7]
*δ*_*d*_	Recovery rate of infected dogs	0.21 year^−1^	Estimated
*γ*	Released rate from infected dogs	9.7 year^−1^	[7]
*μ*_*x*_	Death rate of EEs	1 year^−1^	[8]
*c*_*h*_	Disinfection-induced EE mortality rate	10 year^−1^	Assumed
*Λ*_*l*_	Recruitment rate of livestock	54.33 × 10^4^ year^−1^	Estimated
*β*_*l*_	Infection rate of livestock by ingesting EEs	7.4 × 10^−8^ year^−1^	[7]
*ε*	Fraction of home-slaughtered livestock	0.189	Estimated
*μ*_*l*_	Natural death rate of livestock	0.152 year^−1^	[9]
*Λ*_*h*_	Recruitment rate of humans	1.03 × 10^4^	[29]
*β*_*h*_	Infection rate of humans by ingesting EEs	4.2 × 10^−11^ year^−1^	[7]
*ω*	Reciprocal of human incubation period	1/14 year^−1^	[7]
*μ*_*h*_	Natural death rate of humans	0.0139 year^−1^	Estimated
*δ*_*h*_	Recovery rate of humans	0.041 year^−1^	Estimated
*u*_1_(*t*)	Effectiveness of home slaughter inspection	0–1	Assumed
*u*_2_(*t*)	Effectiveness of anthelmintic treatment	0–1	Assumed
*u*_3_(*t*)	Effectiveness of environmental disinfection	0–1	Assumed
*u*_4_(*t*)	Effectiveness of health education	0–1	Assumed

## Data Availability

The authors confirm that the data supporting the findings of this study are available within the article.

## Appendix

### A. Proof of Theorem 2

The Jacobian matrix of model (1) evaluated at *E*_*dfe*_ is obtained by

(A.1) $$\begin{array}{c} J=\left(\begin{array}{c} \begin{array}{cccccccc} -\mu_{d} & \delta_{d}u_{2} & 0 & 0 & -\frac{\left(1-u_{1}\right)\varepsilon \beta_{d}\Lambda_{d}}{\mu_{d}} & 0 & 0 & 0\\ 0 & -\left(\mu_{d}+\delta_{d}u_{2}\right) & 0 & 0 & \frac{\left(1-u_{1}\right)\varepsilon \beta_{d}\Lambda_{d}}{\mu_{d}} & 0 & 0 & 0\\ 0 & \gamma & -\left(\mu_{x}+c_{h}u_{3}\right) & 0 & 0 & 0 & 0 & 0\\ 0 & 0 & -\frac{\beta_{l}\Lambda_{l}}{\varepsilon +\mu_{l}} & -\left(\varepsilon +\mu_{l}\right) & 0 & 0 & 0 & 0\\ 0 & 0 & \frac{\beta_{l}\Lambda_{l}}{\varepsilon +\mu_{l}} & 0 & -\left(\varepsilon +\mu_{l}\right) & 0 & 0 & 0\\ 0 & 0 & -\frac{\left(1-u_{4}\right)\beta_{h}\Lambda_{h}}{\mu_{h}} & 0 & 0 & -\mu_{h} & 0 & \delta_{h}\\ 0 & 0 & \frac{\left(1-u_{4}\right)\beta_{h}\Lambda_{h}}{\mu_{h}} & 0 & 0 & 0 & -\left(\omega +\mu_{h}\right) & 0\\ 0 & 0 & 0 & 0 & 0 & 0 & \omega & -\left(\mu_{h}+\delta_{h}\right) \end{array} \end{array}\right). \end{array}$$

Then, the corresponding characteristic polynomial is

(A.2) $$\begin{array}{c} P\left(\lambda \right)=\left(\lambda +\mu_{d}\right)\left(\lambda +\mu_{h}\right)\left(\lambda +\varepsilon +\mu_{l}\right)\left(\lambda +\mu_{h}+\delta_{h}\right)\left(\lambda +\omega +\mu_{h}\right)\left(\lambda^{3}+a_{2}\lambda^{2}+a_{1}\lambda +a_{0}\right), \end{array}$$

where

(A.3) $$\begin{array}{c} \begin{array}{c} a_{0}=\left(\varepsilon +\mu_{l}\right)\left(\mu_{d}+\delta_{h}u_{2}\right)\left(\mu_{x}+c_{h}u_{3}\right)\left(1-R_{0}^{3}\right),\\ a_{1}=\left(\varepsilon +\mu_{l}\right)\left(\mu_{d}+\delta_{h}u_{2}\right)+\left(\mu_{d}+\delta_{h}u_{2}\right)\left(\mu_{x}+c_{h}u_{3}\right)+\left(\varepsilon +\mu_{l}\right)\left(\mu_{x}+c_{h}u_{3}\right),\\ a_{2}=\left(\varepsilon +\mu_{l}\right)+\left(\mu_{d}+\delta_{h}u_{2}\right)+\left(\mu_{x}+c_{h}u_{3}\right). \end{array} \end{array}$$

Let *Q*(*λ*) = *λ*^3^ + *a*_2_*λ*^2^ + *a*_1_*λ* + *a*_0_. It is evident from (A.3) that there are *a*_1_ > 0 and *a*_2_ > 0. If *ℛ*_0_ < 1, then *a*_0_ > 0. Furthermore,

(A.4) $$\begin{array}{c} a_{1}a_{2}-a_{0}=\left[\mu_{l}+\left(\mu_{d}+\sigma u_{2}\right)\right]\left[a_{1}+{\left(\mu_{x}+c_{h}u_{3}\right)}^{2}\right]+\mu_{l}\left(\mu_{d}+\sigma u_{2}\right)\left(\mu_{x}+c_{h}u_{3}\right)R_{0}^{3}>0. \end{array}$$

Using Routh–Hurwitz conditions [23], all roots of *Q*(*λ*) have negative real parts. Then, it is clear that all roots of *P*(*λ*) have negative real parts. Therefore, the disease-free equilibrium *E*_*dfe*_ is locally asymptotically stable when *ℛ*_0_ < 1. By contrast, *Q*(0) = *a*_0_ < 0 if *ℛ*_0_ > 1. Since $\underset{\lambda ⟶+\infty }{\lim}Q\left(\lambda \right)=+\infty$, there must be a positive root of *Q*(*λ*) from the Intermediate Value Theorem. So, *E*_*dfe*_ is unstable if *ℛ*_0_ > 1.

The article "Stability Analysis and Optimal Control Strategies of an Echinococcosis Transmission Model" was published in 2022. Journal: Comput Math Methods Med.

### B. Proof of Theorem 3

It is worth noting that the first five equations of model (1) are independent of the last three equations of model (1). So, consider the first five equations of model (1) as a subsystem:

(B.1) $$\begin{array}{c} \left\{\begin{array}{c} {\dot{S}}_{d}=\Lambda_{d}-\left(1-u_{1}\right)\varepsilon \beta_{d}S_{d}I_{l}-\mu_{d}S_{d}+\delta_{d}u_{2}I_{d},\\ {\dot{I}}_{d}=\left(1-u_{1}\right)\varepsilon \beta_{d}S_{d}I_{l}-\mu_{d}I_{d}-\delta_{d}u_{2}I_{d},\\ \dot{X}=\gamma I_{d}-\mu_{x}X-c_{h}u_{3}X,\\ {\dot{S}}_{l}=\Lambda_{l}-\beta_{l}S_{l}X-\varepsilon S_{l}-\mu_{l}S_{l},\\ {\dot{I}}_{l}=\beta_{l}S_{l}X-\varepsilon I_{l}-\mu_{l}I_{l}. \end{array}\right. \end{array}$$

Let (*S*_*d*_(*t*), *I*_*d*_(*t*), *X*(*t*), *S*_*l*_(*t*), *I*_*l*_(*t*)) be any solution of model (B.1) in Γ. This implies that *I*_*d*_(*t*) ≤ *Λ*_*d*_/*μ*_*d*_, *I*_*l*_(*t*) ≤ *Λ*_*l*_/(*ε* + *μ*_*l*_) for all *t* ≥ 0. Define a Lyapunov function as follows:

(B.2) $$\begin{array}{c} L\left(I_{d},X,I_{l}\right)=I_{d}+\frac{\mu_{d}+\delta_{d}u_{2}}{\gamma }X+\frac{\left(1-u_{1}\right)\varepsilon \beta_{d}\Lambda_{d}}{\mu_{d}\left(\varepsilon +\mu_{l}\right)}I_{l}. \end{array}$$

Then, the derivative of *ℒ* along the solutions of model (B.1) yields

(B.3) $$\begin{array}{c} \frac{dL}{dt}={\dot{I}}_{d}+\frac{\mu_{d}+\delta_{d}u_{2}}{\gamma }\dot{X}+\frac{\left(1-u_{1}\right)\varepsilon \beta_{d}\Lambda_{d}}{\mu_{d}\left(\varepsilon +\mu_{l}\right)}{\dot{I}}_{l}=\left(\left(1-u_{1}\right)\varepsilon \beta_{d}S_{d}-\frac{\left(1-u_{1}\right)\varepsilon \beta_{d}\Lambda_{d}}{\mu_{d}}\right)I_{l}+\left(\frac{\left(1-u_{1}\right)\varepsilon \beta_{d}\beta_{l}\Lambda_{d}}{\mu_{d}\left(\varepsilon +\mu_{l}\right)}S_{l}-\frac{\mu_{d}+\delta_{d}u_{2}}{\gamma }\left(\mu_{x}+c_{h}u_{3}\right)\right)X\leq \left(\frac{\left(1-u_{1}\right)\varepsilon \beta_{d}\beta_{l}\Lambda_{d}}{\mu_{d}\left(\varepsilon +\mu_{l}\right)}\frac{\Lambda_{l}}{\left(\varepsilon +\mu_{l}\right)}-\frac{\mu_{d}+\delta_{d}u_{2}}{\gamma }\left(\mu_{x}+c_{h}u_{3}\right)\right)X=\frac{\mu_{d}+\delta_{d}u_{2}}{\gamma }\left(\mu_{x}+c_{h}u_{3}\right)\left(R_{0}^{3}-1\right)X. \end{array}$$

Therefore, $\dot{ℒ}<0$ if *ℛ*_0_ < 1 and *X* > 0. Moreover, $\dot{ℒ}=0$ when *ℛ*_0_ < 1 and *X* = 0. As a consequence, the only invariant set satisfying $\dot{ℒ}=0$ is *E*_*dfe*_ when *ℛ*_0_ < 1. By Lasalle's invariance principle [24], the disease-free equilibrium *E*_*dfe*_ is globally asymptotically stable if *ℛ*_0_ < 1.

Now, consider the last three equations of model (1). From above, it has $\underset{t⟶\infty }{\lim}X\left(t\right)=0$ if *ℛ*_0_ < 1. So, it could be deduced that $\underset{t⟶\infty }{\lim}E_{h}\left(t\right)=0$. Furthermore, $\underset{t⟶\infty }{\lim}I_{h}\left(t\right)=0$ and $\underset{t⟶\infty }{\lim}S_{h}\left(t\right)=\Lambda_{h}/\mu_{h}$ could be derived. Thus, *E*_*dfe*_ is globally asymptotically stable for model (1) when *ℛ*_0_ < 1.

The article "Stability Analysis and Optimal Control Strategies of an Echinococcosis Transmission Model" was published in 2022. Journal: Comput Math Methods Med.

### C. Proof of Theorem 4

Since ${\dot{S}}_{d}+{\dot{I}}_{d}=\Lambda_{d}-\mu_{d}\left(S_{d}+I_{d}\right)$, and ${\dot{S}}_{l}+{\dot{I}}_{l}=\Lambda_{l}-\left(\varepsilon +\mu_{l}\right)\left(S_{l}+I_{l}\right)$, it implies that $\underset{t⟶\infty }{\lim}\left(S_{d}+I_{d}\right)=\Lambda_{d}/\mu_{d}$ and $\underset{t⟶\infty }{\lim}\left(S_{l}+I_{l}\right)=\Lambda_{l}/\left(\varepsilon +\mu_{l}\right)$. So the long-term dynamical behaviors of *S*_*d*_(*t*) and *S*_*l*_(*t*) could be replaced by *Λ*_*d*_/*μ*_*d*_ − *I*_*d*_(*t*) and *Λ*_*l*_/*μ*_*l*_ − *I*_*l*_(*t*), respectively. Consider the subsystem of model (1) as follows:

(C.1) $$\begin{array}{c} \left\{\begin{array}{c} {\dot{I}}_{d}=\left(1-u_{1}\right)\varepsilon \beta_{d}S_{d}I_{l}-\mu_{d}I_{d}-\delta_{d}u_{2}I_{d},\\ \dot{X}=\gamma I_{d}-\mu_{e}X-c_{h}u_{3}X,\\ {\dot{I}}_{l}=\beta_{l}S_{l}X-\varepsilon I_{l}-\mu_{l}I_{l}. \end{array}\right. \end{array}$$

Let

(C.2) $$\begin{array}{c} \Delta =\left\{\left(I_{d},X,I_{l}\right)\in {\mathbb{R}}_{+}^{3}:I_{d}\leq \frac{\Lambda_{d}}{\mu_{d}},X\leq \frac{\gamma \Lambda_{d}}{\mu_{d}\left(\mu_{x}+c_{h}u_{3}\right)},I_{l}\leq \frac{\Lambda_{l}}{\varepsilon +\mu_{l}}\right\}. \end{array}$$

The dynamics of model (C.1) can be focused on Δ since Γ is positively invariant for model (C.1). The method in [25] is adopted to explore the global stability of model (C.1). Define

(C.3) $$\begin{array}{c} h\left(v\right)=\left(\begin{array}{c} h_{1}\left(v_{1},v_{2},v_{3}\right)\\ h_{2}\left(v_{1},v_{2},v_{3}\right)\\ h_{3}\left(v_{1},v_{2},v_{3}\right) \end{array}\right)=\left(\begin{array}{c} -\left(\mu_{d}+\delta_{d}u_{2}\right)v_{1}+\left(1-u_{1}\right)\varepsilon \beta_{d}\left(\frac{\Lambda_{d}}{\mu_{d}}-v_{1}\right)v_{3}\\ -\left(\mu_{x}+c_{h}u_{3}\right)v_{2}+\gamma v_{1}\\ -\left(\varepsilon +\mu_{l}\right)v_{3}+\beta_{l}\left(\frac{\Lambda_{l}}{\varepsilon +\mu_{l}}-v_{3}\right)v_{2} \end{array}\right). \end{array}$$

Then, *h* : ℝ_+_^3^ ↦ ℝ_+_^3^ is a continuously differential map. It thus has *h*(0) = 0, and *h*_*i*_(**v**) ≥ 0, *i* = 1, 2, 3, for all **v** ∈ Δ when *v*_*i*_ = 0. Furthermore, *∂h*_*i*_/*∂v*_*j*_ ≥ 0, *i* ≠ *j*, for **v** ∈ Δ, so that *h* is cooperative on Δ.

For *p* ∈ (0, 1) and **v** ∈ Δ, it has

(C.4) $$\begin{array}{c} h_{1}\left(pv_{1},pv_{2},pv_{3}\right)=-\left(\mu_{d}+\delta_{d}u_{2}\right)pv_{1}+\left(1-u_{1}\right)\varepsilon \beta_{d}\left(\frac{\Lambda_{d}}{\mu_{d}}-pv_{1}\right)pv_{3}\geq -\left(\mu_{d}+\sigma u_{2}\right)pv_{1}+\left(1-u_{1}\right)\beta_{d}\left(\frac{\Lambda_{d}}{\mu_{d}}-v_{1}\right)pv_{3}=ph_{1}\left(v_{1},v_{2},v_{3}\right). \end{array}$$

Similarly, it could be shown that *h*_*i*_(*pv*_1_, *pv*_2_, *pv*_3_) ≥ *ph*_*i*_(*v*_1_, *v*_2_, *v*_3_), *i* = 2, 3. So *h* is strictly sublinear on Δ.

The article "Stability Analysis and Optimal Control Strategies of an Echinococcosis Transmission Model" was published in 2022. Journal: Comput Math Methods Med.

By computing *Dh*(**v**) = (*∂h*_*i*_/*∂v*_*j*_)|_1≤*i*,*j*≤3_, it leads to

(C.5) $$\begin{array}{c} Dh\left(v\right)=\left(\begin{array}{ccc} -\left(\mu_{d}+\delta_{d}u_{2}\right)-\left(1-u_{1}\right)\varepsilon \beta_{d}v_{3} & 0 & \left(1-u_{1}\right)\varepsilon \beta_{d}\left(\frac{\Lambda_{d}}{\mu_{d}}-v_{1}\right)\\ \gamma & -\left(\mu_{x}+c_{h}u_{3}\right) & 0\\ 0 & \beta_{l}\left(\frac{\Lambda_{l}}{\varepsilon +\mu_{l}}-v_{3}\right) & -\left(\varepsilon +\mu_{l}\right)-\beta_{l}v_{2} \end{array}\right). \end{array}$$

Then, *Dh*(**v**) is irreducible on **v** ∈ Δ because |*Dh*(**v**)| ≠ 0. A straightforward computation shows that

(C.6) $$\begin{array}{c} Dh\left(0\right)=\left(\begin{array}{ccc} -\left(\mu_{d}+\delta_{d}u_{2}\right) & 0 & \left(1-u_{1}\right)\varepsilon \beta_{d}\frac{\Lambda_{d}}{\mu_{d}}\\ \gamma & -\left(\mu_{x}+c_{h}u_{3}\right) & 0\\ 0 & \beta_{l}\frac{\Lambda_{l}}{\varepsilon +\mu_{l}} & -\left(\varepsilon +\mu_{l}\right) \end{array}\right). \end{array}$$

Then, the characteristic polynomial of *Dh*(0) is

(C.7) $$\begin{array}{c} Q\left(\lambda \right)=\lambda^{3}+a_{2}\lambda^{2}+a_{1}\lambda +a_{0}, \end{array}$$

where *a*_0_, *a*_1_, and *a*_2_ are known from (B.1). Then, *a*_0_ < 0 when *ℛ*_0_ > 1. According to the proof process of Theorem 3, there must exist a positive root of *Q*(*λ*). Therefore, *s*(*Dh*(0)) = max{Re*λ* : *Q*(*λ*)} > 0. From Corollary 3.2 in [25], there are $\underset{t⟶\infty }{\lim}I_{d}\left(t\right)=I_{d}^{*}$, $\underset{t⟶\infty }{\lim}X\left(t\right)=X^{*}$, and $\underset{t⟶\infty }{\lim}I_{l}\left(t\right)=I_{l}^{*}$. Furthermore, $\underset{t⟶\infty }{\lim}S_{d}\left(t\right)=S_{d}^{*}$ and $\underset{t⟶\infty }{\lim}S_{l}\left(t\right)=S_{l}^{*}$.

When *ℛ*_0_ > 1, the limiting system of the last three equations in model (1) is

(C.8) $$\begin{array}{c} \left\{\begin{array}{c} {\dot{S}}_{h}=\Lambda_{h}-\left(1-u_{4}\right)\beta_{h}S_{h}X^{*}-\mu_{h}S_{h}+\delta_{h}I_{h},\\ {\dot{E}}_{h}=\left(1-u_{4}\right)\beta_{h}S_{h}X^{*}-\omega E_{h}-\mu_{h}E_{h},\\ {\dot{I}}_{h}=\omega E_{h}-\mu_{h}I_{h}-\delta_{h}I_{h}. \end{array}\right. \end{array}$$

It is evident that model (C.8) is linear. By computing the eigenvalues of the linear model (C.8), it could be shown that (*S*_*h*_^∗^, *E*_*h*_^∗^, *I*_*h*_^∗^) is locally asymptotically stable. Therefore, (*S*_*h*_^∗^, *E*_*h*_^∗^, *I*_*h*_^∗^) is globally asymptotically stable. According to [26], it concludes that the endemic equilibrium *E*_*ee*_ of model (1) is globally asymptotically stable.
